This article has been retracted.

# Effect of Zhuyun I Recipe Capsule Enema on the Immune Microenvironment of the Endometrium during Implantation Window in Rats

**DOI:** 10.1155/2022/4746121

**Published:** 2022-10-07

**Authors:** Hang Zhou, Pei Guo, Pengfei Zeng, Zhixing Yin, Li Yan, Jinzhu Huang, Yi Wang, Juan Li, Wanting Xia, Yang Wang, Chang Liu, Qian Zeng

**Affiliations:** ^1^Department of Gynecology, Chengdu University of Traditional Chinese Medicine, Chengdu, Sichuan, China; ^2^Department of Pathology, Hospital of Chengdu University of Traditional Chinese Medicine, Chengdu, Sichuan, China; ^3^Department of Gynecology, Hospital of Chengdu University of Traditional Chinese Medicine, Chengdu, Sichuan, China; ^4^Department of Gynecology, Xinan Gynecological Hospital, Chengdu, Sichuan, China; ^5^Department of Gynecology, Zhengzhou Third People's Hospital, Chengdu, Sichuan, China

## Abstract

**Background:**

Preterm birth is the leading cause of neonatal death, and there are no effective clinical means for the prevention and treatment of spontaneous preterm birth, mainly because the mechanism for labor initiation has not been fully elucidated.

**Objective:**

The effect of enucleation with Zhuyun I Recipe Capsule enema (ZRC) on the maternal-fetal interface microenvironment in SD rats with kidney deficiency and blood stasis.

**Methods:**

In this study, poor endometrial tolerance was induced by hydroxyurea and epinephrine in SD rats with kidney deficiency and blood stasis type of endometrium, and gavage with norethindrone (estradiol) or Bamboo Rhythm No.1 formula. HOXA10 mRNA levels were measured by qPCR. In addition, the expression of IL-6, VEGF, TGF–*β*, and IGFBP-1 in the uterus was detected by IHC and ELISA.

**Results:**

Hydroxyurea- and epinephrine-induced PER was associated with low levels of HOXA10 in the endometrium and reduced levels of IL-6, TGF-*β*, VEGF, and IGFBP-1 in the endometrium. These were abolished by ZRC and Progynova treatment compared to PER rats, resulting in a dramatic increase in the levels of HOXA10 mRNA, IL-6, TGF-*β*, VEGF, and IGFBP-1 proteins.

**Conclusions:**

ZRC improves metaplasticization of endometrial stromal cells and promotes angiogenesis in rats with kidney deficiency and blood stasis. The moderate dose of kidney tonic to promote blood circulation method is superior in promoting angiogenesis, facilitating the establishment and maintenance of pregnancy, limiting trophoblast invasion of metaplasia, reducing miscarriage, and improving pregnancy rate.

## 1. Introduction

The World Health Organization (WHO) estimated in 2013, based on globally available health data, that one in four (25%) couples living in developing countries with a normal desire to have children fail to meet their fertility needs, with female infertility accounting for about one in two of these cases [1, 2]. The latest 2015 guidelines of the American Society for Reproductive Medicine (ASRM) define infertility as the failure of a couple of reproductive age to conceive successfully when they have lived together for more than 1 year, have normal sexual intercourse, and do not use any contraception [3, 4]. For women unilaterally, infertility is the inability to conceive and absence of a full-term delivery despite a pregnancy [5]. From pregnancy to childbirth, women bear more responsibility and stress, both in terms of the vertical line of time spanning the length and the horizontal line of physical burden. With the rise of equal rights for men and women, women are increasingly involved in social production activities and share the cost of living of the family, which inevitably generates more interest, psychological and environmental pressures, plus the fact that Chinese traditional culture is born from Confucianism, which emphasizes the idea of peace as the most important thing, and preaches that “if you don't tolerate a small amount, you will make a big mistake.” The traditional Chinese culture is based on Confucianism, which emphasizes the idea of harmony and promotes the virtues of “if you don't tolerate a little, you'll make a big mistake,” “if you tolerate, you'll get help,” and “a gentleman doesn't argue,” and the two schools of Buddhism and Taoism, which have a common influence on the cultural foundation. There are also related theories such as “the way of heaven is not contentious but good at winning, not saying anything but good at responding” and “of the six degrees and ten thousand actions, patience is the first” [6, 7]. These ideas and statements may have rarely been systematically studied or passively inculcated, but in the trajectory of an individual's growth from childhood to adulthood, there were moments and scenes where he or she was imbued with these ideas, such as the example of elders who taught by themselves. The strong cultural factors may lead Chinese women to have difficult thoughts such as “not good enough to say, afraid to say, unwilling to say” after stress arises, and no effective stress relief mechanism is formed [8]. As a result, gynecological diseases such as infertility occur.

If we think about infertility from a woman's perspective, we should divide the problem into two stages: one is the inability to conceive normally, and the other is the inability to deliver a healthy, viable fetus after pregnancy. Specifically, there are a series of complex, precise, and coordinated physiological processes, including the delivery of good-quality oocytes from the dominant follicle, the movement of the egg in the pelvis and fallopian tube, the swimming of sperm in the reproductive tract, the meeting of sperm and egg to exchange chromatin to form a fertilized egg, the coordination of the embryonic oogenesis progress with the endometrial tolerance, the positioning of the embryonic follicle for adhesion and implantation, the invasion of trophoblast cells, and the normal development of the blastocyst and fetus. The key intersection separating infertility from infertility is at the stage of blastocyst implantation (localized adhesive implantation), or the window of implantation [9, 10]. The endometrial implantation window is a relatively short period of time when the embryo and the intrauterine microenvironment are highly coordinated, synchronized, and unified, partially overlapping with the concept of endometrial tolerance, which simultaneously emphasizes that the role of the embryo cannot be ignored [10].

Kidney deficiency and blood stasis are common syndrome types of infertility [11]. Clinically, the prescription of the effect of Zhuyun I Recipe Capsule enema can achieve ideal results in patients with failed in vitro fertilization-embryo transfer (IVF-ET), kidney deficiency, and blood stasis. Although there are studies on the correlation between laminin and infertility, abnormal expression of adhesion molecules based on kidney deficiency and blood stasis models has not been observed and explained. Although the rectal route has higher bioavailability and reduced hepatic metabolic burden than the oral and force-feeding routes, it has rarely been used in infertility-related animal studies. Therefore, this paper focuses on the effects of the Zhuyun I Recipe Capsule enema prescription on endometrial metaplasia in rats with kidney deficiency and blood stasis models on day 8 of pregnancy and factors related to TGF-*β*, IL-6, and VEGF at the gestational-fetal interface, and explores the possible mechanisms of its role in theoretical support for pregnancy.

## 2. Material and Method

### 2.1. Ethics Statement

The scheme of the animal experiment was approved by the institutional and local animal care and use committees from the Hospital of the Chengdu University of TCM (#2019DL006).

### 2.2. Animal Study

SPF female SD rats (*n* = 36, 5-week-old, 220–240g) from Kunming Laboratory Animal Center were kept in polypropylene cages with sawdust bedding at room temperature with 50% humidity, 12/12 light/dark cycle, and free access to food or water.

After acclimatization, 36 rats were randomly separated into six groups (*n* = 6)^3^. Control rats received 0.9% saline. Rats of H-A (hydroxyurea-adrenaline)-treated group received hydroxyurea (9CO63D05) at a dose of 400 mg/kg daily orally for 9 days, and adrenaline (1710201) at a dose of 0.3 mg/Kg subcutaneously at day 4 to establish the poor endometrial receptivity (PER). Positive control rats (Progynova group) received Progynova (512306042) at a dose of 0.02 mg/kg daily orally for 9 days^4^. In this experiment, the drug dose of SD rats was compared with that of adults (weight: 50 kg). According to the conversion method of drug use dose between rats and humans in “pharmacological experimental methods,” the equivalent dose ratio of the two was 0.018^3^. The formula was as follows: the clinical dose of humans was set as *χ* mg/kg, and the dose conversion of SD rats was as follows:

(1) $$\begin{array}{c} \text{Dosage for }rats\frac{\chi mg/kg*\;50kg\;}{0.2Kg}*0.018=4.5÷\frac{mg}{kg}. \end{array}$$

In ZRC treatment groups, increasing concentrations of TCM were enema (Patent No: ZL20141039113.7) to rats for 10 days at low, middle, and high doses at 8.21, 16.43, and 32.86 g/kg·BW, respectively, each day in the morning (Figure 1). Zhuyun No.1 prescription's composition, proportion, origin, and preparation of the drug are shown in Table 1. Distilled water was used for preparing drugs. Zhuyun No.1 prescription was provided by our hospital. The enema fixator and enema procedure of rats are shown in Figures 1(a) and 1(b).

On day 10, female and male rats (2 : 1) were put together. The day seeing vaginal plugs was set as pregnancy day 1 and drugs were provided until day 5. Then, rats were killed for ELISA assay and checking implantation status^5^. Both implantation rate and average number of embryos were sharply decreased in PER rats compared to controls, indicating the successful PER establishment. The intervention flow chart of the whole experiment is shown in Figure 1(c).

### 2.3. Procedure of Rat Enema Drug Administration

After 1 week of acclimatization and observation of the vital status and general signs of the adult female rats of SPF class SD, the rats were weighed and numbered after confirmation of no obvious pathology. Pull up vertically (avoid lifting from the end to cause damage); place in the supine position, exposing the lower abdomen; assistant No. 2 synchronous preparation: raise the sacrococcygeal area of the rat about 40°, use a 5ml enema syringe to inject the liquid into the rat's anus about 8cm. After pushing, take out the syringe with one hand, and immediately clamp the anus with a sterilized wooden clip with the other hand, keep it for 20 minutes, and put it into the cage, as shown in Figure 1.

### 2.4. Procedure of Smear Operation to Monitor Morphological Changes in Endometrium

Operate in the following acid-base staining sequence: 95% alcohol fixation ⟶ hematoxylin staining ⟶ tap water wash ⟶ 1% hydrochloric acid differentiation ⟶ tap water wash ⟶ 1% eosin staining ⟶ tap water wash ⟶ xylene solution. The operation time of each step was as follows: 5 min, 7 min, 5–10s, 5s, 5–10s, 1 min, 5–10s, and 5 min; and remove the slide to control the excess liquid. Then, place the slide in a position with good air convection to dry naturally and place it under the microscope for observation. (Points to note: when the cotton swab is applied to the slide, firstly, the front and back of the slide should be distinguished, and the frosted side, which is convenient for writing the number in the hand, should be the front side, which is conducive to the last step of microscopic observation (reducing the time for distinguishing the front and back sides); secondly, the force should be appropriate so that the secretion is transferred to the slide without destroying the cells, and the overlap of the different spreads on the same slide should be minimized to reduce the stacking of cells. Because the nuclear staining solution has certain volatility and the degree of cell density and sparseness varies, the specific staining time can be adjusted according to the specific situation. The staining time can be adjusted according to the specific situation).

### 2.5. Scanning Electron Microscopy Observation

Acicular cells (number and morphology): SEM preparation procedure: fixation with osmic acid for 2 hours at 4°C; rinse with distilled water twice (8 minutes each); stepwise dehydration twice in 50%, 70% and 90% ethanol (each 8 minutes); 100% alcohol dehydration at room temperature for 10 minutes; isoamyl acetate = 1 : 1, 3 : 7, 1 : 9, each dehydration for 10 minutes; pure isovaleric acid dehydration for 10 minutes; hexamethyldimethylamine drying 10 minutes”. Ultrathin sections were made; acinar cell count: 12 fields of view were randomly selected from each sample to observe acinar cells according to the Rebecca method, and the lumen surface of endometrial epithelial cells was selected according to the range of acinar cells for scoring: 0 Score: no acinar cells; 1 score: < 25%; 2 score: 25%-50%; 3 score > 50%, then the scores were statistically analyzed.

### 2.6. Enzyme-Linked Immunosorbent Assay (ELISA)

The uterine tissue was homogenized with five volume lysis buffer and centrifuged at 800 g for 15 min. The supernatant containing the cytoplasmic part was stored in a refrigerator at −80°C for the detection of indicator proteins. IL-6 kit (ab9324, Abcam, USA), TGF-*β* ELISA kit, VEGF ELISA kit, and IGFBP1 ELISA kit (F16921, F171720, and F15791, WESTING Co. Ltd, CHN) were used to detect the protein of uterine homogenate.

Preparation of standard solution: take eight 1.5 ml centrifuge tubes, add 900 *μ*l sample diluent into the first tube, and add 500 *μ l* sample diluent into the second-to-eighth tubes. Add 100 *μ*l of a standard solution of 10 *μ*g/ml into the first tube, place it on the vortex mixer, and then suck out 500 *μ*l with the sampler and move it to the second tube. In this way, repeated double dilution was performed, and 500 *μ*l was aspirated from the seventh tube and discarded. The eighth tube was blank control. Dilute with 1 : 20 double distilled water, add 100 *μ*l of plasma to each well, mix well, wash 4–6 times at 37°C for 40 min, dry on filter paper, add 50 *μ*l double distilled water and primary antibody to each well except blank, mix well, wash plate at 37°C for 20 min, add 100 *μ*l enzyme-labeled antibody, wash plate at 37°C for 10 min, and add 100 ul substrate working solution at 37°C in dark light. After 15 min, 100 UL of the solution was added to stop mixing, and OD450 was recorded. Taking 1000, 500, 250, 125, 62.5, 31.2, 15.6, and 0 ng/ml as abscissa and OD value as ordinate, the standard curve was drawn with software. The content of each index was calculated according to the OD value of the sample.

### 2.7. Immunohistochemical (IHC) Staining

Uteri were fixed in paraformaldehyde. After slicing, dewaxed sections were put into the dyeing vat, 3% methanol H2O2 was used for 15 min, and PBS was used for washing three times (8 min each). The slices were immersed in 0.01 M citrate buffer solution, boiled in the microwave oven, and then the power was cut off. The procedure was repeated one time 5 min later. After cooling, PBS was washed twice for 5 min each time. The blocking liquid of goat serum was dripped and kept at room temperature for 20 minutes. Rabbit anti-rat IL-6 polyclonal antibody (ab9324, Abcam, USA), rabbit anti-rat TGF-*β* polyclonal antibody (abs15221, Absin, CHN), rabbit anti-rat VEGF polyclonal antibody (abs131208, Absin, CHN), and rabbit anti-rat IGFBP-1 polyclonal antibody (abs136650, Absin, CHN) were added to the groups with different indexes. Add biotinylated second antibody at 37°C for 30 min; wash three times with PBS water for 5 min each time; use DAB color reagent kit, mix the reagent, drop it on the slice, develop color at room temperature, control the reaction time under the microscope, generally about 2 min, and wash with distilled water. The specimens were lightly counterstained with hematoxylin, dehydrated, transparent, mounting slides with neutral gum for light microscope examination. A Ba200 digital trinocular camera system (McCurdy Industrial Group Co., Ltd.) was used to capture 3 fields of view for the processes of dehydration, trimming, embedding, sectioning, staining, and sealing.

### 2.8. Relative Real-Time PCR (qRT-PCR) Assay

After thawing the tissue on ice, pour out the preservation solution, add 1 ml Trizol into the EP tube to extract DNA from uterine tissue, confirm the quality of nucleic acid, reverse transcription, add 90 *μ*l referee water to dilute, add corresponding primers, using GAPDH as an internal reference, and the annealing temperature is 54°C. Amplification conditions as follows: 94°C 3 min, 30 cycles, and extension at 72°C for 10 min. Levels of Ang-1, Ang-2, and Tie-2 were measured by SYBR green method: HOXA10 F5′-TGCATATTTGGAATGCGCCG-3'and R5′-CCAAGAATCTCGCTGGGGTT-3′.

### 2.9. Statistical Analyses

SPSS 22.0 was applied for data analysis. If data not only meet the normal distribution but also conform to the homogeneity of variance, the one-way ANOVA and LSD test are used to compare the data among groups. If the data conform to the normal distribution but the variance is not uniform, thanes' T2 test is used for comparison among groups after ANOVA analysis. The data in the following table are all expressed by means ± standard deviation (*x* ± *s*). If data are not normally distributed, Mann–Whitney *U* test was adopted to analyze the comparison between the groups.

## 3. Results

### 3.1. Condition of Uterus and Endometrium

The wet weight of the uterus and the index of uterine organs of model rats were sharply decreased compared to normal controls (Figure 2). However, compared to model rats, the uterus wet weight and uterine organ index of low-, heavy-, and high-dose ZRC groups and the control group were significantly higher, especially in ZRC medium-dose group (*P* < 0.05). Under the light microscope, the endometrium of the blank group was covered with intact epithelium, well-developed, sufficient epithelial cells, abundant blood vessels, regular glands, large glandular cavity, and loose interstitial arrangement, showing spindle shape; in the model group, the endometrium was covered with thin, poorly developed, less epithelial cells, fewer glands, narrowed glandular space, not rich blood vessels, dense stroma, and some stromata were compact. The development was not synchronized. In ZRC low-, medium-, and high-dose groups, the endometrial epithelia showed an increasing trend. The epithelial cells were evenly arranged in a long columnar shape, with abundant glands. The glandular cavity was round or oval, with abundant blood vessels and even and loose stroma. The normal group had abundant villi, with mononuclear cells on the surface of the villi, round and full, as mature pinopodes; and the model group had few villi on the surface of the endometrium, with serious destruction, and a small amount of pinopodes expression in the developing stage. The level of pinopodes in the ZrC group was higher than that in the model rats, especially in the middle- and high-dose groups, and the pinopode expression in the middle-dose group tended to be mature. The number of pinopodes in the positive group was also more than that in the model rats, but slightly less than the drug group, for the developing pinhole, which tended to be mature.

### 3.2. IL-6 Expression in Endometrial Tissue in Treated Rat

The IL-6 expression in uterine tissue in PER H-A rats was sharply downregulated compared to normal controls (Figure 3). Compared to PER H-A rats, Progynova or TCM drastically upregulated IL-6 levels in uterine tissue (*P* < 0.05).

The TGF-*β* expression in endometrial PER H-A rats was sharply downregulated compared to controls (Figure 4). Compared to PER H-A rats, Progynova or ZRC at middle or high doses drastically upregulated TGF-*β* in endometrial. No significant difference was found between low-dose ZRC and model rats.

### 3.3. VEGF Levels

Compared to controls, PER H–A rats have lower uterine VEGF levels (Figure 5), which were sharply upregulated by Progynova or ZRC. Compared to PER-Progynova, high-dose ZRC drastically upregulated uterine VEGF.

### 3.4. IGFBP-1 Levels

PER H-A rats exhibited significantly lower uterine IGFBP-1 than controls (Figure 6), which were sharply upregulated by Progynova or ZRC treatment.

### 3.5. HOXA10 Levels

Compared to controls, PER H-A rats had a significantly low HOXA10 mRNA, which was sharply upregulated by Progynova. However, ZRC (8.21 g/kg) drastically upregulated HOXA10 mRNA, compared to Progynova treatment (Figure 7).

## 4. Discussion

The specific pathogenesis of endometriosis (EM) is still unclear and has been inconsistently understood by researchers over the years, including the implantation theory, the somatic epithelial metaplasia theory, and the induction theory [12]. The classical implantation theory proposed by Sampson has been accepted by many researchers, and the main routes of transmission include retrograde flow, lymphatic and venous dissemination, and medical implantation, among which the most recognized route of transmission is retrograde flow [13]. With a deeper understanding of EM, it was found that the explanation of the mechanism of EM pathogenesis by menstrual reflux seems to be one sided because it cannot explain multiple as well as extrapelvic EM, and fails to explain why only 10%–15% of so many women with common menstrual reflux develop EM [14].

In recent years, it has been proposed that EM is an immune disorder [15, 16]. The ectopic endometrial tissue in normal women acts as a foreign body that induces immune cells in the peritoneal fluid and stimulates an immune response, which results in the removal of endometrial tissue or cells that reflux with menstrual blood. In contrast, EM patients develop immune tolerance to their own organism, resulting in ectopic endothelial tissue or cells failing to be removed by evading surveillance by the immune system and thus implanting and growing in the pelvic abdomen, forming ectopic lesions.

It is increasingly recognized that angiogenesis is an important link in the development of EM, endometrial angiogenesis disorders may be an important pathological basis for EM pathogenesis and an important feature of EM, and the survival and growth of EM lesions are dependent on abundant blood supply [17]. The presence of a large number of blood vessels in the peritoneal and ectopic endothelial tissues surrounding EM was seen by laparoscopy and histopathology, respectively [18]. It was found that the in situ endothelium of EM patients was rich in vascular growth factors, and their vascular growth potential was stronger than that of the in situ endothelium of healthy women [19].This result is consistent with the “in situ endothelium” determinism proposed by Academician Lang Jinghe, who believes that ectopic endothelium can only become a lesion in the pelvic and abdominal cavity after the “three-part process” of adhesion, invasion, and blood vessels [20].

Enema is a traditional method of treating diseases by inserting drugs into the anus or intestines, and it has unique advantages in treating infertility. Firstly, the location of the uterus (womb and adnexa) is adjacent to the rectum, and the drug can act directly on the uterus and the ramus; secondly, the drug is warm but not hot, which can warm up the blood vessels; meanwhile, “the lung and the large intestine are adjacent to each other,” and the drug can be delivered to the whole body through the action of “all the veins converge in the lung.” According to this study, the formula of “activating the blood circulation around the rectum” avoids blood stagnation in the kidneys and clinical efficacy is better. Rectal administration can reduce the stimulation of drugs to the gastrointestinal tract and improve the bioavailability of drugs; the absorption pathway is mainly absorbed by the middle rectal vein, inferior vein, and anal vein, accounting for 50%–70% of drug absorption; rectal administration significantly reduces the first-pass elimination effect of the liver and increases the local blood concentration; meanwhile, a small amount of drugs enter the liver from the superior rectal vein and participate in the general circulation after metabolism. Many clinical reports have shown that enemas can improve blood concentration, viscosity, and coagulability, improve endometrial blood supply, promote pelvic circulation, and increase clinical pregnancy rates in patients with infertility/IVF-ET failure [20]. See Figure 8.

Currently, an increasing number of studies have found that growth factors and cytokines play an important role in maternal-fetal interactions during embryo implantation [21]. On the one hand, it is known that the endometrium makes inflammatory cytokines. On the other hand, cyclic changes in inflammatory cytokine expression in the uterus are associated with the proliferative and secretory phases, especially during the implantation window. Although some studies have shown that cytokines are regulated by steroid hormones such as estradiol and progesterone, some experimental studies have shown that autocrine and paracrine cytokines regulate local steroid hormones [22]. Thus, the balance of the inflammatory immune microenvironment at the embryo-maternal interface is indispensable for successful embryo positioning, adhesion, and implantation.

During the early stages of embryonic development, angiogenesis is the most essential condition for meconium and embryo implantation. The vascular endothelial growth factor is the most potent mitogenic factor that promotes blood vessel growth, stimulates angiogenesis, and maintains vessel wall permeability and integrity. A study [23] has shown that reduced or no expression of VEGF in localized areas can lead to poor angiogenesis, abnormal differentiation, and infiltration of trophoblast cells, resulting in miscarriage or implantation failure.

By comparing the morphology of metaphase on the 8th day of pregnancy, it was found that kidney deficiency and blood stasis could inhibit endometrial metaphase. Low, medium, and high doses of Zhuyun I Recipe Capsule improved methylation of endometrial stromal cells and promoted angiogenesis in rats with kidney deficiency and blood stasis. The middle dose of Zhuyun I Recipe Capsule was better than other groups in promoting angiogenesis, which was beneficial to the establishment and maintenance of pregnancy, limiting the invasion of trophoblast into the metaplasia, reducing abortion, and improving the pregnancy rate. It has a bidirectional regulating effect on ovulation, reduces the increase in blood viscosity caused by cold stimulation and blood clotting, can regulate reproductive endocrine, improve ovarian function, regulate analgesia and vasodilatory function of patients, and restore normal ovarian function. Study [24]showed that the warming and activating effect of Zhuyun I Recipe Capsule can promote the growth of endometrium and follicles and facilitate the discharge of follicles. The study [25] concluded that Bamboo Zhuyun I Recipe Capsule can promote ovulation and transport sperm, thus achieving the purpose of treating infertility.

Thus, from the analysis of the formula and modern pharmacology, as well as from the experimental and clinical efficacy of Zhuyun I Recipe Capsule for EM, it can effectively treat EM by enhancing immunity (tonifying the kidney) and improving hemodynamics (resolving blood stasis).

### 4.1. Problems and Prospects

The shortcomings of this experimental study: firstly, the estrogen level of rats is much lower than that of humans, and there may be some limitations when extrapolating the results from animal models to humans; secondly, in the rat autologous endograft mapping over, considering the large workload, different personnel were involved in the suturing, which caused some errors in the experiment. In combination with this experiment, we will conduct clinical and in vitro cellular experiments in the future to further explore the specific mechanism of action of Zhuyun I Recipe Capsule on EM with kidney deficiency and blood stasis. Second, in the future EM modeling process, we will learn from the experience of this experiment and adopt a clear division of labor to achieve uniformity and minimize avoidable errors due to handling factors.

## Figures and Tables

**Figure 1:** Note: (a) Rat enema fixator: it is composed of a fixing strap, soft pad, and frame plate. (b) Rat enema administration process: the rats were placed in the prone position and bound to the fixator by hook loop; and the operator stroked the abdomen of rats along the colon and stimulated the anus of rats so that the rats could discharge the feces of the lower intestinal tract as much as possible and make them empty, which is conducive to the retention and absorption of liquid medicine. Next, it was confirmed that the feces were no longer excreted, the operator raised the sacrococcygeal region of rats about 40° and injected the liquid into the anus of rats about 8 cm with a 5 ml enema syringe, and pushed it slowly and evenly. After pushing, one hand was used to take out the syringe, while the other hand immediately used the sterilized wooden clip to clamp the anus, keeping it for 20 minutes, and putting it into the cage; (c) Experimental intervention flowchart.

**Figure 2:** Note (a) wet weight of the uterus and the index of the uterine organs. (b) Expression of endometrial morphology (HE,×200) and pinocytosis morphology (SEM,×3000) in treated rats: (a) Controls; (b) Hydroxyurea + Adrenaline; (c) Progynova; (d) ZRC (8.21 g/kg·BW); (e) ZRC (16.43 g/kgv·BW); and (f) ZRC (32.86 g/kg·BW). (c) There were significant differences in the mean ± standard deviation of the endocytosis score under the electron microscope among the groups.

**Figure 3:** IL-6 levels in endometrial tissue. Note: (A) IHC staining of IL-6: (a) Normal controls; (b) H-A; (c) Progynova; (d) ZRC (8.21 g/kg·BW); (e) ZRC (16.43 g/kgv·BW); and (f) ZRC (32.86 g/kg·BW). (B) Levels of IL-6 by ELISA. TGF-*β* expression in endometrial tissue in treated rat.

**Figure 4:** Levels of TGF-*β*. Note: (A) TGF-*β* levels in rat endometrial tissues: (a) Normal control; (b) H-A; (c) Progynova; (d) ZRC (8.21 g/kg); (e) ZRC (16.43 g/kg); and (f) ZRC (32.86 g/kg). (B) TGF-*β* in rat endometrial tissues is shown by ELISA.

**Figure 5:** Levels of VEGF. Note: (A) VEGF levels in rat endometrial tissue: (a) Normal control; (b) H-A; (c) Progynova; (d) ZRC (8.21 g/kg BW); (e) ZRC (16.43 g/kg·BW); and (f) ZRC (32.86 g/kg·BW). (B) VEGF levels shown by ELISA.

**Figure 6:** Levels of IGFBP-1. Note: (A) Endometrial GFBP-1 levels: (a) Normal control; (b) H-A; (c) Progynova; (d) ZRC (8.21 g/kg); (e) ZRC (16.43 g/kg); and (f) ZRC (32.86 g/kg). (B) IGFBP-1 levels are shown by ELISA.

**Figure 7:** (a) HOXA10 concentration curve and initial concentration curve. Note: (B) Relative mRNA expression in endometrium: (a) Normal control; (b) H-A; (c) Progynova; (d) ZRC (8.21 g/kg BW); (e) ZRC (16.43 g/kg·BW); and (f) ZRC (32.86 g/kg·BW).

**Figure 8:** Mechanism of enema in TCM.

**Table 1:** Composition and source of Zhuyun I prescription.

Product name	Scientific name	Production unit	B.N.	Place of production	Proportion of weight
TuSizi	*Cuscuta chinensis lam.*	Sichuan Guoqiang Herbal Pieces Co., Ltd	19030104	Sichuan	3
FuPenzi	*Rubus idaeus* L.	Sichuan BaiCaoYuan Pharmaceutical Co., Ltd	190401	Zhejiang	2
GouQizi	*Lycium chinense Mill.*	Sichuan Qianyuan Herbal Pieces Co., Ltd	191201	NingXia	2
DanShen	*Salvia miltiorrhiza Bunge.*	Sichuan Jiuweige Herbal Pieces Co., Ltd	191901	Sichuan	2
XuDuan	Dipsacales	Sichuan Heyi Natural Pharmaceutical Co., Ltd	19071704	Sichuan	4
Shanzha	*Crataegus pinnatifida Bunge*	Sichuan Hengkangyuan Pharmaceutical Co., Ltd	191001	Shanxi	3
ShanYao	*Dioscorea oppositifolia* L.	Sichuan Guoqiang Herbal Pieces Co., Ltd	19080105	Henan	3
SiGualuo	*Luffa cylindrica*	Sichuan Herbal Pieces Co., Ltd	190614	Sichuan	3

## Data Availability

The data used to support the findings of this study can be obtained from the corresponding author upon reasonable request.

## References

[1] Achache H., Revel A. (2006). Endometrial receptivity markers, the journey to successful embryo implantation. *Human Reproduction Update*.

[2] Ying Li, Zhu R. (2007). Studies on the expression of integrin *β*1 and laminin in endometrium of infertile patients and normal early pregnancy decidual tissue. *Journal of Mathematical Medicine*.

[3] Sun J. (2001). *Animal Experiment Method*.

[4] Qianyi F., He D., Xu L. (2014). Establishment of a rat model of kidney deficiency, blood stasis and endometrial receptivity. *Henan Traditional Chinese Medicine*.

[5] Peng Z., Hai-Bin K., Physiology D. O. (2013). *Endometrial Decidualization Model and its Application Research Progress*.

[6] Wanting X., Yanmei Z., Ying Z. (2017). Curative effect of assisted reproduction technology by Traditional Chinese Medicine multi-channel interventional therapy on 95 cases of in vitro fertilization and embryo transfer failure. *Journal of Traditional Chinese Medicine*.

[7] Hongxiang X. (2011). Clinical observation on endometriosis-induced infertility treated by herbal enema. *Journal of Practical Traditional Chinese Medicine*.

[8] Salker M., Teklenburg G., Molokhia M. (2010). Natural selection of human embryos:impaired decidualization of endometrium disables embryo-maternal interactions and causes recurrentpregnancy loss. *PLoS One*.

[9] Li S., Zhao F., Liu R. (2007). Expression of matrix metalloproteinase-9 and laminin and pregnancy outcome in abortion model. *Shanxi Medical Journal*.

[10] Shi Y., Wu L., Mu G. (2017). Effects of erjianyu decoction and modified Recipe on the expression of integrin *ανβ*3, SCF mRNA and HOA-10 mRNA in mouse endometrium. *Chinese Journal of Traditional Chinese Medicine*.

[11] Tabibzadeh S., Kong Q. F., Babaknia A., May L (1995). Progressive rise in the expression of interleukin-6 in human endometrium during menstrual cycle is initiated during the implantation window. *Human Reproduction*.

[12] Dziekoński M., Zmijewska A., Franczak A., Kotwica G., Czelejewska W., Okrasa S. (2015). The expression of mRNAs for opioid precursors in endometrium of cyclic and early pregnant pigs; effects of IL-1*β*, IL-6 and TNF*α*. *Journal of Animal and Feed Sciences*.

[13] Godkin J. D., Doré J. J. (1998). Transforming growth factor beta and the endometrium. *Reviews of Reproduction*.

[14] Lennard S. N., Stewart F., Allen W. R. (1995). Transforming growth factor-*β*1 expression in the endometrium of the mare during placentation. *Molecular Reproduction and Development*.

[15] Kim M. R., Park D. W., Lee J. H. (2005). Progesterone-dependent release of transforming growth factor-beta1 from epithelial cells enhances the endometrial decidualization by turning on the Smad signalling in stromal cells. *MHR: Basic science of reproductive medicine*.

[16] Yi X. J., Jiang H. Y., Lee K. K. H., O W. S., Tang P. L., Chow P. H. (1999). Expression of vascular endothelial growth factor (VEGF) and its receptors during embryonic implantation in the golden hamster (*Mesocricetus auratus*). *Cell and Tissue Research*.

[17] Kaczmarek M. M., Kiewisz J., Schams D., Ziecik A. (2009). Expression of VEGF-receptor system in conceptus during peri-implantation period and endometrial and luteal expression of soluble VEGFR-1 in the pig. *Theriogenology*.

[18] Shangwei L., Zongjian T., Ziyan H. (2002). *Expression of IGFBP-1 and IGFBP-2 in Endometrium and Their Relationships with Serum Progesteron during Peri-Implantation in Rat*.

[19] Zhu L. H., Sun L. H., Hu Y. L. (2013). *β*PCAF impairs endometrial receptivity and embryo implantation by down-regulating *β*3-integrin expression via HOXA10 acetylation. *Journal of Clinical Endocrinology and Metabolism*.

[20] Gordon J. A. R., Hassan M. Q., Saini S. (2010). Pbx1 represses osteoblas togenesis by blocking HOXA10-mediated recruitment of chromatin remodeling factors. *Molecular and Cellular Biology*.

[21] Gaide Chevronnay H. P., Selvais C., Emonard H., Galant C., Marbaix E., Henriet P. (2012). Regulation of matrix metalloproteinases activity studied in human endometrium as a paradigm of cyclic tissue breakdown and regeneration. *Biochimica et Biophysica Acta, Proteins and Proteomics*.

[22] Salleh N. (2014). Diverse roles of prostaglandins in blastocyst implantation. *The Scientific World Journal*.

[23] Seckl J. R., Meaney M. J. (2004). Glucocorticoid programming. *Annals of the New York Academy of Sciences*.

[24] Yin K. J., Deng Z., Hamblin M., Zhang J., Chen Y. E. (2011). Vascular PPAR*δ* protects against stroke-induced brain injury. *Arteriosclerosis, Thrombosis, and Vascular Biology*.

[25] Hwang J. S., Kim H. J., Kim G. (2014). PPARdelta reduces abdominal aortic aneurysm formation in angiotensin II-infused apolipoprotein E-deficient mice by regulating extracellular matrix homeostasis and inflammatory. https://pubmed.ncbi.nlm.nih.gov/24698256/.

